The article "Optimal Loading Height: A Practical Research of Drop Jump from Biomechanics" was published in 2022. Journal: J Healthc Eng.

# Optimal Loading Height: A Practical Research of Drop Jump from Biomechanics

**DOI:** 10.1155/2022/4173639

**Published:** 2022-03-15

**Authors:** Zehao Tong, Wenjia Chen, Hang Xu, Feng Zhai

**Affiliations:** ^1^College of Physical Education, China University of Mining and Technology, Xuzhou, Jiangsu, China; ^2^Department of Medical Imaging, Xuzhou Medical University, Xuzhou, Jiangsu, China

## Abstract

Plyometrics training is paid great attention by coaches and researchers because of its significant effect on the level of lower limb explosive athletes. Many coaches and reseachers use the biomechanical methods to determine optimal loading height for drop jump. The researchers' findings in determining optimal loading height were highly biased and were not applied effectively to training practices. This paper reviews the development process of optimal loading height in deep-jump training, combs the relevant concepts and biomechanical mechanisms of optimal loading height in deep-jump training, and looks forward to the future research.

## 1. Introduction

Plyometrics training has always been an important topic among coaches and researches. The drop jump is a core part of this training program. In the plyometrics training, biomechanical methods are applied to determine the optimal loading height for drop jump. It is an important approach to maximize the training effects, prevent sports injury, and realize evaluation and individualized training for the high-level athletes. In the movement of drop jump, the drop height when the average power output and reactive strength reach a peak is called as the optimal loading height [1, 2]. Besides, the optimal loading height in broad sense covers the drop jump drop height under the maximum values of indicators such as vertical counteracting force, utilization rate of lower limb resilience, and rebound height. Researches examine the relevancy between related indicators of optimal loading height (such as average power and reactive strength) and the sports performance on the basis of determining the optimal loading height of drop jump and select the loading height of drop jump according to the aforesaid relevancy, which can make the research findings applied in sports training more effective.

Drop jump (DJ) in plyometrics training is defined as an exercise of applying a force on the ground with the body weight of athletes, while optimal loading height of drop jump is confirmed to show a significant correlation with the biomechanical indicators collected from the drop jump. The optimal loading height of related drop jump training covers two aspects, namely, average power output and jump height when the reactive strength reaches a peak. Among the academic community, the ability of muscles to quickly absorb centrifugal pull and later generate centripetal force in the stretch-shorten cycle (SSC) is referred to as reactive strength [1]. The average power output is defined as the output of power within a unit of time [3]. Since the landing buffer in the process of drop jump and the later stage of stretch and jump, the muscles have finished a quick coupling from eccentric contraction to centripetal contraction, so drop jump is a typical movement in the SSC. Numerous literature studies have proven that reactive strength and average power output can be used to effectively evaluate the ground pressing duration and jump height during the stage of stretch in drop jump [1, 4]. Therefore, reactive strength and average power output are closely related with the generation of optimal loading height of drop jump. Though researchers have reached a consensus on the significant impact of optimal loading height for DJ on low limb explosive power, the researchers' findings in determining the optimal loading height are highly biased. It has gradually become a focus of the researchers to improve the sports performance through an effective application of optimal loading height.

## 2. Method

In this study, all the evidence was collected from Web of Science. By the “topic search” in Web of Science, The keywords searched include “Plyometrics Training,” “Drop Jump,” “Stretch Shorten Cycle,” “Reactive Strength Index,” “Average Power Output,” etc.

## 3. Origin and Development of Optimal Loading Height for DJ

In 1968, Werschoshanskij initially defined the scope of drop jump loading height (0.9–2.2 m) and confirmed the optimal loading height for DJ at 0.75 m. According to the research, when the height of drop jump is 0.75 m^6^, it has the best training effect on lower limb explosive power. Later, other researchers carried out further researches and experiments based on the preliminary scope defined by Werschoshanskij and determined the optimal loading height for DJ based on the average power output. Scholars Robber et al [7] discovered that the average power output is maximum when the height for DJ is 0.2–0.4 m. When the height reaches 0.6 m, the vertical counteracting force during the stretch of lower limbs will reach a peak. They argued that the drop height for DJ shows a positive correlation with the vertical counteracting force and average power output, and there is an optimal loading height of vertical counteracting force and average power output when the drop height is 0.2–0.6 m^7^. Later, Lee et al. [6] reached a different conclusion. The experimental results indicated that when the drop height for DJ is 0.36 m, the vertical counteracting force reaches the peak, and the loading height for DJ under the maximum average power output is 0.12 m^8^. This discovery challenged the viewpoint of Bobbert et al. that vertical counteracting force and average power output will increase with the rise of loading height for DJ, which indicates that only under a reasonable loading height can muscles achieve the maximum vertical counteracting force and average power output. With the enriching of related research theories and popularization of plyometrics training, the US National Strength and Conditioning Association (2008), based on the conclusions of earlier researchers, suggested that exercisers should control the height scope for DJ training in 41–107 cm to avoid sports injury [7]. Later, Matic et al. verified the speculation of scholars such as Bobbert and found in studies that the loading height with the maximum average power output when the drop height of drop jump is 0.2–0.6 m. Based on the distinctive differences between the excellent group (0.62 m) and the ordinary group (0.32 m) with maximum strength in the heights of maximum average power output, they discovered that the maximum strength had a significant impact on the optimal loading height of average power output [2]. Giminiani and Petricola, based on an experiment of varying DJ heights at 0.2–0.6 m among male athletes, discovered that the maximum average power output [6] could be achieved when the DJ loading height was at 0.4 m.

### 3.1. Maximum Average Power Output

According to the relevant past studies on determining the DJ drop height of maximum average power output, the earlier studies (1968) focused on determining the optimal loading height of common DJ. Due to factors such as immature measurement means and shortage of theoretical reference, the drop height of maximum average power output was relatively high as recorded in earlier literatures (0.75 m). The primary reason is that according to the law of free falling body in mechanics, the movement for DJ is seen as an ideal model of free falling body converting the gravitational potential energy of human body into kinetic energy, which deems that the drop height and the average power output are always in a directly proportional relationship, but neglects the physiological property of muscles, and cannot control the DJ loading height within a small scope (0.9–2.2 m) [7]. Later, sports injury is caused to athletes due to the improper loading height in DJ training. In order to ensure the safety during training, researchers (1969–1994) kept decreasing the height scope for DJ training (0.2–0.6 m) and the loading height of maximum average power output had declined significantly (0.12–0.3 m) [7]. With the maturing of biomechanics measurement means and deepening of theoretical research, many studies had reduced the control of the DJ height scope. After the original dynamic signals were collected with the 3D dynamometric platform, the optimal loading height for DJ of the individuals (0.4–0.47 m) was accurately determined through quadratic polynomial regression analysis [9].

Since scholars such as Werschoshanskij proposed the theory of reactive strength [7, 10–12] and researchers such as Woo conducted in-depth research on the trainability of reactive strength through animal experiments [13–13], many researchers have made relevant explorations to determine the optimal loading height for DJ based on the indicators of reactive strength [13, 12, 14]. Byrne et al. formally defined optimal loading height and confirmed for the first time the optimal loading height of lower limb reactive strength at 0.3 m^16^. The optimal loading height (0.24 m) for the DJ reactive strength index determined by Barr and Nolte was consistent with the earlier research result, who discovered that reactive strength at the DJ height of 0.24 m showed a high reliability in the evaluation of 60-meter running performance (*p* < 0.001) [15]. Later, Byrne et al. determined the new optimal loading height of reactive strength (0.5 m) once again. The author discovered that the reactive strength at the DJ height of 0.5 m showed a relatively high reliability in evaluating the distance of throwing sport (ICC = 0.87), which can be taken as a basis for throwers to select materials [16]. Campillo et al. determined the optimal loading height for DJ of individual athletes with maximum reactive strength (0.2–0.4 m) and applied the optimal loading height of individuals in the seven-week training intervention that followed, which had significantly increased the speed of the athletes in the 20-meter acceleration running (*P* < 0.001,*d* = 0.25), which once again proved that the loading height for DJ at the maximum reactive strength showed a high reliability in evaluating the performance of short sprints [17]. However, Healy et al. questioned the reliability of the reactive strength for DJ in evaluating the performance of short sprints. The author believed that the indicators of reactive strength for DJ showed no significant correlation with the short sprint [4]. Boullosa adopted a warmup with the optimal loading height for DJ for athletes with reactive strength in the experiment. After triggering the Post-Activation Potentiation (PAP), it had shortened the time of 1,000-meter running (pre = 165.3 s, post = 162.4 s) and the time of the first 400 meters (pre = 40.3 s, post = 38.8 s) for male athletes. The performance of male athletes in the 1,000-meter running had not improved significantly, and the performance of female athletes in the 1,000-meter running had declined. For factors such as these, it had failed to prove in depth the reliability of the optimal loading height of reactive strength in evaluating the performance of 1,000-meter running [18].

### 3.2. Reactive Strength

Compared with average power output, researchers are less biased in the determination of optimal loading height of reactive strength. The theory on reactive strength indicators and relevant indicator formula has given rise to this trend. Academically, the reactive strength index is defined as the ratio between jump height and the length of supporting duration [1]. Reactive strength ratio is defined as one between the lengths of duration of flight and supporting duration [19]. Obtaining a higher rebound height or a shorter supporting duration in the DJ test is a precondition to maximize the reactive strength index and ratio. A series of earlier studies indicated that it will significantly lengthen the supporting duration after falling onto the ground if the drop height for DJ is too high [9, 20]. Therefore, researchers (2010–2018) usually adopted a relatively small scope for DJ drop height to test the optimal loading height of reactive strength (0.24–0.3 m), but the optimal loading height determined in some literature studies (2016) was higher (0.5 m), mainly because of differences of experimental subjects in such aspects as gender [21], sport events [22], and age [23]. A lot of literature studies has proven the high reliability of reactive strength during DJ in the evaluation of short sprints and throwing. Therefore, the reactive strength has gradually become an important indicator for the effective evaluation of the muscle performance during the stretch-shorten cycle.

## 4. Application of Optimal Loading Height for Drop Jump

Among the various means of plyometrics training, DJ is an important component of special physical training for athletes as well as a detection means for the lower limb explosive power of athletes. The determining of optimal loading height for DJ has prominent values to athletes in such aspects as physical training, personality assessment, and sports injury prevention. Therefore, relevant studies on optimal loading height for DJ are not only focused on typical stretch-shorten cycle sports such as sprint and jump but also in special physical training such as rugby, volleyball, and soccer. Though a lot of literature has reported the optimal loading height for DJ in different sports, only a very few of the researchers have applied the optimal loading height in training practice and achieved distinctive effects, which mainly cover intervention to DJ training with optimal loading height with reactive strength and improved the performance of 20 m and 1,000 m running. Earlier related conclusions still need to be further verified with intervention experiments later.

Various sport events selected and applied the optimal loading height for DJ. Byrne et al. [17] discovered based on reactive strength indicators that the optimal loading height of throwers was 0.5 m. Barr and Nolte [15] discovered that the height for maximum power output of high-level women's rugby sport was 0.24 m. Zehao Tong et al. clarified that male high jumper also has the optimal height of reactive strength index (0.45 m) at four heights (0.3–0.75 m)^44^.The literature report by researchers such as Campillo [17] showed that the height for maximum reactive strength of soccer players in DJ training was 0.2–0.4 m. In addition, on the loading heights for DJ among volleyball players, the researchers had put forward different viewpoints. Peng et al. based on the indicators of maximum vertical counteracting force on knee and ankle joints determined that the optimal loading height for DJ of male volleyball players was 50–100% of the CMJ height [24]. This indicates that relevant researches on ball players were mainly about skill-dominant competitions in the same court and net competitions focused on special physical training of the accelerating capacity over a short distance, which is related with the high reliability of optimal loading height reactive strength in DJ for evaluating the accelerating performance over a short distance.

Currently, the relevant studies on the determining of optimal loading height for DJ are mainly focused on biomechanics theoretical research, biomechanical characteristics analysis of athletes, detection of lower limb explosive power of athletes, and the impact factors of reactive strength on sports performance. There are three stages in the exploration of optimal loading height for DJ, namely, determining the common optimal loading height, determining the optimal loading height of sport items (groups), and determining the indicators of optimal loading height for individuals. In determining relevant indicators of DJ height, the researchers showed a trend of diversification. That is, there are great differences among related indicators of optimal loading height determined for various sport items. The relevant indicators of short stretch-shorten cycles (with a coupling duration <0.17 s) represented by high jump and long jump are, respectively, the utilization rate of lower limb resilience and the maximum duration of flight. In the case of long stretch-shorten cycles represented by 100-meter sprint (with a coupling duration >0.17 s), the optimal loading height for DJ is determined through the indicators of average power output and reactive strength. In the case of volleyball with a short stretch-shorten cycle, the optimal drop height for DJ is explored based on the indicators of stretch duration and vertical counteracting force [24]. The forming of this trend may be related with the differences of athletes of various sport items in their take-off techniques and nerve accommodation strategies during DJ and the selection of indicators with the highest association with sports performance in the DJ.

## 5. Biomechanical Mechanism of Optimal Loading Height for Drop Jump

The exact biomechanical mechanism for typical stretch-shorten cycle sports such as DJ has been quite clear; that is, in the mechanical model, the SSC is defined as a fast coupling where the series elastic matter in the muscle-tendon complex is passively pulled centrifugally to store a lot of elastic potential energy, which is unleashed through centripetal shortening [25–27].

However, researchers have not reached a consensus on how the optimal loading height for DJ is formed. That is, the forming of optimal loading height may be subject to various factors. On the one hand, neural feedforward and muscle preactivation play an important role in the SSC [28], which has been supported by the EMG experiment results of many studies [29–31]. Within an appropriate scope of loading height, in Figure 1, the H-reflex of soleus and M-wave will increase significantly until the optimal loading height reaches the peak. In the case of DJ finished at a height too high, the reduction of La afferent neural feedback of *α* motor neuron leads to the significant decline of H-reflex and M-wave of soleus (13.9 ± 7.6%; 8.3 ± 6.5%; *p* < 0.01) [21, 30, 31]. In addition, in the SSC, the H-reflex level of soleus is also subject to objective factors such as temperature [32], duration [33], and the stiffness of landing surface [34]. Within an appropriate scope of drop height, the muscle stretch load will increase with the increase of drop height. The regulation of reflex muscles such as muscle spindle will enhance the preactivation of muscle-tendon complex at the excited lower limbs, which is manifested as the higher stiffness of muscle-tendon complex and accumulation of more elastic potential energy [35]. When it exceeds the optimal loading height, due to the protection from upper spinal nerves, the muscle-tendon complex is protected from a high-load impact and the nerves are adapted to the strategy, the inhibition flow of muscle spindle will lower the preactivation of muscles [9], which is mainly manifested as lower stiffness of the muscle-tendon complex^43^, the significant extension of supporting duration and the loss of the stored elastic potential energy.

On the other hand, the regulation of muscle stiffness by neural feedback and myotatic reflex in the SSC cannot be ignored. If the drop height of DJ is too high, the muscle-tendon complex will be prone to a bigger impact load and a faster traction. The inhibition effect of the Golgi complex will weaken the myotatic reflex of muscle-tendon complex, lower the activation level around the ankle joint muscle, and lower the stiffness of ankle joint [27], which can protect the muscle-tendon complex from injury under a high stress^43^.

## 6. Conclusions

Though earlier studies have proven the superiority of optimal loading height for DJ in sports injury prevention and improvement of the explosive power training effect, due to the complexity of optimal loading height measurement for individuals and differences in biomechanical parameters among individuals and timeliness, the coaches have failed to apply the regularity of optimal loading height for DJ in the specific physical training of athletes.

Researchers need to study more optimal loading parameters and develop mature and comprehensive training plans for individuals according to the biomechanical indicators and characteristics of the research subjects. The differences among individuals in the training should be monitored with biomechanical technology, and the development of biomechanical technologies should be accelerated to realize individualistic testing and evaluation for the specific physical training of high-level athletes. [6–38].

## Figures and Tables

**Figure 1:** H-reflex for soleus in different drop heights [25]. LH = 30 cm drop height, MH = 50 cm drop height, LH = 70 cm drop height.

## Data Availability

The datasets used and/or analyzed during the current study are available from the corresponding author on reasonable request.
